# The Understanding of Medical Informatics among Dental and Medical Students

**DOI:** 10.1155/2022/5141568

**Published:** 2022-10-05

**Authors:** Sarah M. Allabun

**Affiliations:** Medical Education Department, Medicine College, Princess Nourah bint Abdulrahman University, Riyadh, Saudi Arabia

## Abstract

**Background:**

Current medical care deeply relies on informatics during all stages of patient care, which is significantly enhanced due to its use. The healthcare professional's formation in medical informatics results crucial for their everyday practice. However, healthcare study programs not always provide education about the use of this wide variety of systems, and young professionals find that they need to learn about it over the experience. The aim of this study was to assess the understanding of medical and dental students regarding medical informatics and ICTs.

**Materials and Methods:**

A questionnaire was produced with 3 sections and a total of 24 questions. Students replied to the survey before and after taking the medical informatics course.

**Results:**

A total of 719 students from second year of medical and dental school were recruited for the study between the period of September of 2017-May 2018, September 2018-May 2019, September 2019-May 2020, and September 2020-May 2021. Medical and dental students showed a good level of understanding regarding medical informatics, as well as a good perception of the relevance of ICT learning for the professional practice. Course attendance increased the percentage of students that felt confident of their knowledge about medical informatics. However, most students felt that little or no medical informatics education was lectured at their schools and that the University should adapt the academic program to include it. After taking the course, the student's perception on this matter was improved.

**Conclusion:**

Medical and dental students find medical informatics learning useful for their future professional practice and feel inclined to use it. However, they feel that Universities need to adapt their programs in order to include medical education courses and trainings; partly because they are not completely aware of the use of ICTs that already are established in their courses.

## 1. Introduction

The automation of medical informatics was introduced in the second half of the twentieth century [1]. Medical informatics is the science focusing on storing, acquiring, and using medical data or information in health care facility, frequently applying information technology [2]. This broad subtitle includes the digitalization of patients record (such as electronic medical records (EMR) and digital imaging systems), access to knowledge-based data and clinical decision support systems, and telemedicine. Another term strongly related to this field is evidence-based medicine (EBM) that mainly aims to develop new tools in order to facilitate patient care decision-making [3].

Medical informatics was not usually thought in the institutions or in training sessions. However, currently many training institutions are offering postgraduate degrees in this/related field (computer science or intelligent systems) where students mostly have a medical doctor degree. Furthermore, some programs focus on informatics of a specific medical field including dentistry or nursing for example. Informatics in the field of molecular biology and genomics or as known Bioinformatics is expected to expand dramatically due to the recent infusions of funding from the National Institutes of Health.

Professionals in this domain are expected to be skilled in medical information resources and its access including medical journals, literature databases, medical textbooks, practice guidelines, and the increasing number of “synthesized” evidence-based resources (Cochrane Database). Bioinformatics must also have the ability to navigate in these resources on a specific subject using the correct vocabulary and terms involving the Medical Subject Headings (MeSH) and other full-text resources that are not manually indexed.

Technology evolvement has also reached the dental profession where it is not impossible on a computer to decide treatment options and decision-making of patient's care [4]. Dental informatics is still in its early development phase with promising results in improving care quality at the clinical settings. Unfortunately, dental informatics is not well understood by a large proportion of dentists and how they can be a part of it [5].

For example, dental informatics can be used in diagnosis of oral diseases, e-prescriptions, indications, and contraindication of certain drugs in specific groups of patients and many more, therefore, dentist must be updated to improve their performances. Similar to general healthcare, dental informatics is combining both medicine practice and information technology to improve dental research, education, and treatment choices [5]. Friedman reported in his “fundamental theorem” of informatics that informatics is appropriate when implemented to help professionals perform cognitive responsibilities better yet not to mimic or replace human proficiency [6].

Previous reports showed that the conventional method of record keeping resulted an 11% of repeated laboratory tests with misplaced results, a 30% of undocumented treatment orders, 50% of missing or incomplete medical records, a 35% loss of time of physicians and nurses due to paper work, and almost 20-30% of national healthcare expenses on these paperwork [7].

A previous study reported 90% of dentists have a computer in whom only 25-30% use it during work [8] and very few of them use it to the fullest extent and potential, including paperless patient charts or clinical and therapeutic patient outcomes evaluation [9].

It is important to minimize the gap between dentists and computer utilization in order to enhance its practice, with many innovations including decision support, real-time information diffusion, and continuing edification [10]. In consequence, health professionals also must fully understand health informatics and its applications and evaluation. Dental informatics will help students, faculty, and administrators appreciate how dental informatics can be not only used in patient care and also how can it lift up the state of the art in education and research [4]. Many published articles described dental informatics, yet only little on how to implement it especially in less developed countries.

## 2. Materials and Methods

This study was approved by the Ethics Committee of IRB Registration Number with KACST, KSA: HAP-01-R-059. Students registered for the course of Medical Informatics at third year of bachelor's degree of medical and dental schools were recruited. The course was designed to increase the understanding of medical informatics among healthcare students and to provide skills regarding ICTs.

A questionnaire was produced with 3 sections and a total of 24 questions. Students replied the survey before and after taking the medical informatics course, using a qualitative scale (not confident to extremely confident, not important to extremely important, and no opportunity to frequent opportunity). Items of the survey included if they felt confident about the benefits of learning medical informatics and if they believed that it was important to include it in their curricula. Also, items related to the student's perception of the opportunities' availability to learn about medical informatics were added.

The % of students that answered each question was calculated, and mean % of students each section of the survey was compared. In order to determine if behaviour among medical and dental students was different, separate and joint analysis was performed.

## 3. Results

A total of 719 students from second year of medical and dental school were recruited for the study between September of 2017-May 2018, September 2018-May 2019, September 2019-May 2020, and September 2020-May 2021. A questionnaire was provided to the students during the first and the last lecture of a Medical Informatics Course, to evaluate the understanding of Medical Informatics of medical and dental students. A total of 322 students participated before the course (60.9% from medical school and 39.1% from dental school) and 397 students after the course (67.7% from medical school and 32.3% from dental school).

Students were asked if they thought that communication technologies were beneficial for their practice and for the patient care and if they appreciated its advantages even if it meant that they had to invest time into acquiring skills.

Forty seven % of the students expressed that they felt confident and 13.7% said that they felt very confident about using communication technologies and about knowing its benefits (Table 1). Interestingly, this number ascended to 56.9% and 24.6% accordingly after the students took Medical Informatics course and the percentage of students that did not feel confident changed from 8.4% to 2.5%. Regarding recognizing and understanding of ICT for patient care, medical student showed more confidence before 11.5 ± 23.9 vs. 8.1 ± 17.4 (very confident + confident answers) and after the course 19.4 ± 33.6 vs 9.8 ± 15.9 compared to dental student with better results after taking the course. Medical students were more confident in applying technology and information management tools to support safe processes of care especially after the course (19.9 ± 34.8 after and 10.8 ± 22.4 before). More than 80% of students were more confident in plan and document patient care in an electronic health record.

Most of the students (approximately 80%) believed that learning information technology skills was important, and this perception was almost twice larger among medical students (Table 2). Almost none of the students from neither degrees believed that such learning was not important. Consequently, taking the course did not affect the already good perception about learning information technology skills. However, after taking the course, the proportion of students that believed that using information technologies (question 4, Table 2) were extremely important and important part of their professional practice was increased from 67.1% to 78.6%.

As shown in Table 3, the perception of the students regarding their curricula offering for ICTs learning was increased after taking the course. Mean % of students that believed there were no opportunities during their studying program to learn about ICTs was 21.6% before taking the course, and the proportion decreased to 10.4%, along with an important increase in students that believed there were frequent opportunities to learn ICTs (53% to 70.1%). These improvements were more related to medical students that reflected the same changes, whereas dental students did not exhibit the same behaviour.

## 4. Discussion

It has been proposed that healthcare professional education has been left behind when it comes to medical informatics [11]. Since misuse of electronic records and systems can lead to error, students need to train in a safe learning environment [12]. Applying medical informatics courses during bachelor degree provides skills without any risk. The results of study indicate that dental and medical students from our university have some understanding of medical informatics, understanding that was increased after the students attended medical informatics course. We believe that medical informatics course was, indeed, useful to provide new ICT skills to the students, who felt more confident about their knowledge at the end of the course.

According to our observations, the students exhibited a good basal understanding of the benefits that learning medical informatics provides. It has been reported that medical and dental students from first year are more motivated to learning when multimedia resources and self-directed research activities are the pedagogical conditions [13]. It could be thought that young students include ICTs in their everyday life and that they are aware of its general importance and this could mean that they are more prone to its use not only for learning but also for their future professional practice [13].

As expected, attending medical informatics course was able to increase the number of students who became aware of medical informatics advantages. A report by Cresswell et al. [14] published a teaching program to increase medical informatics knowledge and skills among medical students from John Hopkins University. Their findings indicated that students enhanced their knowledge after taking the course. However, further evaluations indicated that this knowledge was limited after attending the course, implying that students might need training practices in addition to courses. It should be noticed that we have not performed evaluations to assess the students acquired knowledge, and that future studies should contemplate them.

Additionally, our findings showed that medical students appeared to show better understanding of ICTs after taking the course. A previous study showed that 63% of dental students preferred active learning lectures with use of technology over traditional classes, which shows a potential good attitude towards ICTs [15]. Another study indicated that both medical and dental students processed new information in an easier and more effective manner by using mobile devices provided by Helsinki University. The students indicated that their teacher's resistance to use technology devices was, however, a barrier [16]. Furthermore, the dental student's attitude towards mobile learning was shown to be positive in another report [17]. In contrast, a previous study by Abromitis [18] indicated that predoctoral dental students overestimated their abilities regarding biomedical database research. In accordance to these reports, it could be though that both medical and dental students have a good understanding of ICTs, but they might possibly develop different skills related to their own specialty and previous education. Medical students might take more advantage of the course due to a previous acquisition of some skill sets potentially, biomedical database research for example. After attending the course, the students clearly understood that medical informatics is an important aspect of their future professional practice. The study performed among medical students in John Hopkins University showed similar effects [14]. Apparently, healthcare students would need medical informatics courses to become aware of its implications.

The relevance of IT healthcare has been long reported as well as the need of trained healthcare professional users [19–21]. This is supported by many international associations that are creating recommendations to achieve standardized competences [14, 19]. The student's future professional practice and lifelong learning most likely will be guided by these recommendations, and it would be relevant to introduce the contents during bachelor degree courses.

The perception of the students regarding the curricula offering for ICTs learning was increased after taking the course. Research studies have been carried out in order to develop a curriculum that effectively provides medical informatics knowledge and skills [22, 23]. Currently, the International Medical Informatics Association recommendations regarding medical informatics curricula needs include core knowledge and skills, system organization, informatics/computer science, mathematics, and biometry. Our results indicate that students might not be aware of medical informatics learning already available in their schools and that during medical informatics course they may have been able to appreciate it. It could be thought that students might learn some of these aspects included in other courses related to other topics but using ICTs. However, we believe that more studies should be carried out to design appropriate medical informatics curricula that facilitates not only learning and training but also the evaluation of the long term acquired knowledge.

## 5. Limitations of the Study

This study was performed with over 700 recruited students, which is an appropriate sample size representative of the studied population. However, while all the students completed the survey after attending the course, approximately 322 students completed the survey before the course, which could skew the data and, consequently the conclusions regarding the effects on the student's knowledge, attitude, and importance of ICT perception. Also, there was no quantitative evaluation of the student's acquired knowledge, to produce more reliable conclusions based on mean comparisons statistical analysis with quantitative data, such as final tests with marks or employing surveys that allow calculating scores [24]. On the other hand, the program of the course included traditional classes and e-learning classes (online). The blending of the lecture types could introduce heterogeneity and an additional source of variation among the students, given that attitude towards lesson impairments may change among different groups of students and among lessons types.

Moreover, we observed that the medical and dental students considered the course as a general one and not as a training course, as intended to assess knowledge and importance perception of medical informatics, indicating that the program might need modifications in this way and that the perception of it being a general course could falsely affect the results of the study in relation to ICTs. Despite these limitations, the study is valid to evaluate the proposed aims.

## 6. Conclusion

In conclusion, medical and dental students find medical informatics learning useful to their future professional practice and feel inclined to use it. However, they feel that Universities need to adapt their programs in order to include medical education courses and trainings; partly because they are not completely aware of the use of ICTs that already are established in their courses.

## Figures and Tables

**Table 1:** Understanding of the benefits of communication informatics.

I feel confident in my ability to:	Before the course (%)			After the course (%)		
	Dental	Medical	Total	Dental	Medical	Total
(1) Describe the benefits of different communication technologies						
Extremely confident	4	9.6	13.7	8.1	16.5	24.6
Confident	16.5	29.2	45.7	19.3	37.6	56.9
Somewhat confident	15.5	16.8	32.3	4.3	11.7	16
Not confident	3.1	5.3	8.4	0.5	2	2.5
(2) Describe examples of how technology and information management are related to the quality and safety of patient care						
Extremely confident	6.8	13.4	20.2	9.8	23.2	33.1
Confident	20.8	28.6	49.4	19.4	35.1	54.5
Somewhat confident	9	14.9	23.9	2.8	7.8	10.6
Not confident	2.5	4	6.5	0.3	1.5	1.8
(3) Recognize the time, effort, and skill required for computers, databases, and other technologies to become reliable and effective tools for patient care						
Extremely confident	8.1	11.5	19.6	9.8	19.4	29.3
Confident	17.4	23.9	41.3	15.9	33.6	49.5
Somewhat confident	8.7	18.6	27.3	6.6	11.6	18.2
Not confident	5	6.8	11.8	0	3	3
(4) Seek education about how information is managed in care settings before providing care						
Extremely confident	5.9	11.5	17.4	7.6	21	28.6
Confident	18.7	21.2	39.9	19.2	31.6	50.9
Somewhat confident	11.5	19.9	31.5	4.8	12.2	17
Not confident	2.8	8.4	11.2	0.8	2.8	3.5
(5) Apply technology and information management tools to support safe processes of care						
Extremely confident	5	10.8	15.8	9.8	19.9	29.8
Confident	21.4	22.4	43.8	17.7	34.8	52.5
Somewhat confident	10.9	18.3	29.2	4.5	10.9	15.4
Not confident	1.9	9.3	11.2	0.3	2	2.3
(6) Navigate the electronic health record						
Extremely confident	5.3	8.7	14	8.3	16.7	25
Confident	18	17.1	35.1	17.7	33.6	51.3
Somewhat confident	10.9	22	32.9	6.1	13.4	19.4
Not confident	5	13	18	0.3	4	4.3
(7) Employ communication technologies to coordinate care for patients						
Extremely confident	5.3	9.1	14.4	10.1	20.5	30.6
Confident	21.9	23.8	45.6	18.7	33.4	52.2
Somewhat confident	9.4	18.8	28.1	3.5	12.2	15.7
Not confident	2.8	9.1	11.9	0	1.5	1.5
(8) Document patient care in an electronic health record						
Extremely confident	10.9	13	23.9	12.9	27.6	40.5
Confident	21.4	23	44.4	18	29.1	47.1
Somewhat confident	5.3	13.7	18.9	1.3	9.9	11.1
Not confident	1.6	11.2	12.7	0	1.3	1.3
(9) Plan care in an electronic health record						
Extremely confident	8.1	9.9	18	13	24.9	37.9
Confident	19.3	22.4	41.9	16.8	28.8	45.5
Somewhat confident	9.3	16.5	25.8	1.8	11.7	13.5
Not confident	2.2	12.1	14.3	0.5	2.5	3.1
(10) Use information management tools to monitor outcomes of care processes						
Extremely confident	6.2	12.1	18.3	9.6	20.2	29.8
Confident	18	21.4	39.4	17.2	31.6	48.7
Somewhat confident	11.2	16.1	27.3	5.6	12.9	18.4
Not confident	3.7	11.2	14.9	0	3	3
(11) Use high quality electronic sources of health information						
Extremely confident	8.1	11.2	19.3	10.2	23.6	33.8
Confident	17.4	21.5	38.9	17.8	28.7	46.4
Somewhat confident	10.6	16.5	27.1	4.6	11.9	16.5
Not confident	3.1	11.5	14.6	0	3.3	3.3
(12) Protect confidentiality of protected health information in electronic health records						
Extremely confident	10.9	18.7	29.6	12.7	27.3	40
Confident	17.1	22.7	39.9	17.5	30.4	47.8
Somewhat confident	9.3	13.1	22.4	2.3	7.8	10.1
Not confident	1.9	6.2	8.1	0	2	2

**Table 2:** Importance of acquiring information technology skills and relevance to healthcare practice.

It is important to me that:	Before the course (%)			After the course (%)		
	Dental	Medical	Total	Dental	Medical	Total
(1) I seek lifelong learning of information technology skills						
Extremely important	11.4	23.7	35.1	11.1	22.9	34
Important	20.3	26.9	47.2	15.2	31.2	46.4
Somewhat important	6.6	8.9	15.5	5.9	8.8	14.7
Not important	0.9	1.3	2.2	0.5	4.4	4.9
(2) All health professionals seek lifelong learning of information technology skills						
Extremely important	10.2	23.5	33.7	12.1	21.4	33.6
Important	18.7	27	45.7	15	31.3	46.3
Somewhat important	9.8	9.5	19.4	5.7	12.7	18.3
Not important	0.6	0.6	1.3	0	7	7
(3) There are technologies that support clinical decision-making, error prevention, and care coordination available to me in my practice						
Extremely important	12.3	25.3	37.7	11.4	27.7	39.1
Important	19.3	26.3	45.6	16.8	27.7	44.6
Somewhat important	6.6	8.5	15.2	4.1	10.1	14.2
Not important	0.9	0.6	1.6	0.5	1.6	2.1
(4) My profession is involved in the design, selection, implementation, and evaluation of information technology						
Extremely important	10.1	14.9	25	11.3	16.2	27.6
Important	17.7	24.4	42.1	17.8	33.2	51
Somewhat important	7.6	18.7	26.3	3.6	13.9	17.5
Not important	3.8	2.8	6.6	0	15	15

**Table 3:** Opportunities during the curricula program for ICT learning.

In my studying program I had opportunities to:	Before the course (%)			After the course (%)		
	Dental	Medical	Total	Dental	Medical	Total
(1) Use electronic health records in the learning laboratory						
Frequent opportunity	11.1	9.5	20.6	13.7	17.7	31.4
Occasional opportunity	15.6	16.8	32.4	12.9	25.8	38.7
Minimal opportunity	7.3	18.1	25.4	4.1	15.4	19.5
No opportunity	4.8	16.8	21.6	1.5	8.9	10.4
(2) Document care in an electronic health record in the clinical setting						
Frequent opportunity	16.3	10.3	26.6	17.7	21.3	39
Occasional opportunity	12.2	15.6	27.8	12.9	25.1	38
Minimal opportunity	6.6	12.2	18.8	1.5	10.4	11.9
No opportunity	4.4	22.5	26.9	0.3	10.9	11.1
(3) Plan care in an electronic health record in the clinical setting						
Frequent opportunity	13.4	10	23.4	17.5	21	38.5
Occasional opportunity	12.5	12.8	25.3	12.2	25.1	37.2
Minimal opportunity	7.5	15.6	23.1	2.5	10.9	13.4
No opportunity	5.9	22.2	28.1	0.3	10.6	10.9
(4) Use various communication technologies to coordinate care for patients in the clinical setting						
Frequent opportunity	10	9.4	19.4	15.2	22.1	37.3
Occasional opportunity	15	17.2	32.2	12.7	21.8	34.5
Minimal opportunity	10	14.4	24.4	4.6	12.4	17
No opportunity	4.4	19.7	24.1	0	11.2	11.2
(5) Use a database to support patient care						
Frequent opportunity	13.6	10.8	24.4	14.7	22	36.7
Occasional opportunity	15.2	15.8	31	14.4	23.3	37.7
Minimal opportunity	7	14.9	21.8	2.5	12.7	15.2
No opportunity	3.8	19	22.8	0.8	9.6	10.4
(6) See examples of clinical decision making supports and alerts						
Frequent opportunity	10.3	10.6	20.9	12.9	21	33.8
Occasional opportunity	14.7	19.1	33.8	13.6	26.8	40.4
Minimal opportunity	9.1	15.6	24.7	5.1	14.1	19.2
No opportunity	5.3	15.3	20.6	0.8	5.8	6.6
(7) Compare different communication technologies						
Frequent opportunity	5.6	10	15.7	11.1	22.3	33.4
Occasional opportunity	14.4	17.6	32	13.9	25.8	39.7
Minimal opportunity	12.5	17.2	29.8	5.6	14.4	20
No opportunity	6.9	15.7	22.6	1.8	5.1	6.8
(8) See examples of how technology and information management are related to the quality and safety of patient care						
Frequent opportunity	11.3	15.3	26.6	13.4	28.3	41.7
Occasional opportunity	13.8	17.8	31.6	14.9	25	39.9
Minimal opportunity	11.6	15	26.6	3.3	10.3	13.6
No opportunity	2.8	12.5	15.3	0.8	4	4.8

## Data Availability

The data used to support the findings of this study are included within the article.
